# Dexmedetomidine Combined with Low-Dose Propofol Declines Learning and Memory Impairment and Neural Cell Injury in Developing Rats

This article has been retracted.

**DOI:** 10.1155/2022/9543459

**Published:** 2022-05-31

**Authors:** Xiaoxu Yin, Peng Jiang, Jing Li

**Affiliations:** ^1^Department of Anesthesiology, Huizhou Central People's Hospital, Huizhou, Guangdong 516001, China; ^2^Department of Anesthesiology, The Second Affiliated Hospital of Xi'an Medical University, Xi'an, Shaanxi 710038, China

## Abstract

**Background:**

General anesthesia in early childhood may affect all aspects of neurodevelopment, resulting in learning and behavior defects. Therefore, there is an urgent need to find safe anesthetics or put forward more comprehensive anesthesia schemes to solve the negative effects caused by existing anesthetics. The objective of this study is to explore the impact of dexmedetomidine (Dex) incorporated with low-dose propofol (PRO) on learning and memory ability and neural cells in developing rats.

**Methods:**

Eighty SD rats were randomly divided into 4 groups including the Sham group, Lipid group, L-PRO group, and Dex + L-PRO group. After treatment, the spatial learning and memory ability of rats in each group were assessed by the water maze test and the passive avoidance test. The damage of hippocampal tissues was assessed by Nissl staining; the apoptosis, the levels of inflammatory factors, and the level of oxidative stress were measured by Tunel staining, ELISA, and biochemical assays, respectively. Besides, qRT-PCR and Western Blot determined the expression of apoptosis-related proteins, neurotrophic factors, and MAPK signaling pathway-related proteins in the hippocampus.

**Results:**

Compared with the L-PRO group, the Dex + L-PRO group had better spatial learning and memory ability. Administration of Dex and L-PRO greatly alleviated neural cell damage in the hippocampus and decreased the levels of IL-6, IL-1*β*, and TNF-*α*. Besides, it significantly decreased the content of ROS and malondialdehyde (MDA), glutathione (GSH), when up-regulating the levels of IL-10, antioxidant superoxide dismutase (SOD) and BDNF, receptor tyrosine kinase B (TrkB), and neurotrophin-3 (NT-3) related to hearing function and significantly lower activity of MAPK signaling pathway.

**Conclusion:**

Dex combined with low-dose PRO can significantly inhibit inflammation, oxidative stress response, neuronal apoptosis, MAPK signaling pathway activity and promote the secretion of neurokines in hippocampus to reduce neural cell damage and avoid the learning and memory impairment caused by anesthetics in developing rats.

## 1. Introduction

It is reported that millions of children receive anesthesia during surgery or diagnostic procedures each year in the United States [1], and general anesthesia is the most common practice to relieve pain during surgery in most clinical treatments for children [2]. However, anesthesia exposure is noted to lead to neurotoxicity in the developing brain [3]. Moreover, children exposed to anesthetics in the early years showed a higher incidence of brain learning deficits during adolescence [4]. A number of meta-analyses have reported that maternal use of anesthetics may lead to neurotoxicity and neurological damage to the fetus [5]. Receiving general anesthesia at an early age may induce learning and behavioral deficits by affecting various aspects of their neuronal development [6]. DiMaggio et al. found that young children exposed to anesthesia were more than twice as likely to appear behavioral impairment or developmental deficits in their later life, including mental retardation, autism, and language disorders [7]. However, some researchers have pointed out that the harm caused by anesthetics to children may depend on the anesthesia time, frequency of use, and other factors related to the anesthesia regimen. The above findings have raised concerns about the possible nerve damage caused by commonly used anesthetics in pediatrics. Therefore, there is an urgent need to find safe anesthetics or to propose more comprehensive anesthetic regimens to address the negative effects caused by existing anesthetics.

According to different action principles, the commonly used anesthetics and sedatives are currently divided into two categories in clinical practice. Combination with *γ*-aminobutyric acid receptor agonist (GABA) receptor or N-methyl-D-aspartate (NMDA) receptor may strengthen the anesthetic effect, respectively. GABA binders include volatile anesthetic gases, propofol (PRO), barbiturates, etomidate, and chloral hydrate, while NMDA binders include nitrous oxide and ketamine [8]. Because their mechanism of action is similar to the interaction of normal neurotransmission, they may cause adverse effects on neuronal apoptosis and synaptogenesis in the rapidly developing immature brain. However, some researchers have found that dexmedetomidine (Dex), an *α*^2^-adrenergic receptor agonist, is effective and highly selective [9]. Dex can reduce neuronal apoptosis induced by isoflurane and ketamine *in vivo* and *in vitro* [10]. Additionally, with antioxidant and antiapoptotic activities, Dex can produce neuroprotection by up-regulating astrocyte brain-derived neurotrophic factor (BDNF) expression and inhibiting the PI3K/Akt/GSK- 3*β* pathway [11]. Α2-Adrenergic receptor subtype is widely expressed during brain development, and Song et al. found that it mediates the neurotrophic effects of norepinephrine and dendritic growth of cortical neurons during fetal cortical development [12]. Dex often serves as a sedative for children in clinical practice and is considered to be a highly effective and safe adjuvant for anesthetics. Wang et al. found that Dex alleviated hippocampal apoptosis and juvenile cognitive deficits caused by repeated PRO in juvenile rats through the PI3K/Akt/Gsk-3*β* pathway [13]. However, the study by Wang et al. did not involve the effects on neural cells in developing juvenile rats, and there is no study to explore the effects of Dex and PRO on learning and memory ability in juvenile rats. Therefore, the aim of this study was to explore the effects of Dex combined with PRO on nerve injury, learning, and memory ability in developing rats. A rat model of nerve injury was established. And these evidence propose new reflections and methods to solve the harm of anesthesia in children.

## 2. Materials and Methods

### 2.1. Rat Model Construction and Treatment

All the experiments were approved by the Guangdong Experimental Animal Center Ethics Committee. Eighty SD rats on postnatal day 7 (P7) were collected and the animals were randomly divided into four groups (*n* = 20) with similar physiological status, including the Sham group, Lipid group, L-PRO group, and Dex + L-PRO group. Sham group: P7 rats were untreated; Lipid group: P7 rats were injected with lipid emulsion (major adjuvant of PRO solution) via tail vein; L-PRO group: P7 rats were injected with PRO at a dose of 5 mg/kg (H20030115, Sichuan Guorui Pharmaceutical Co., Ltd., Sichuan, China) through the tail vein, followed by maintenance anesthesia at a dose of 30 mg/kg/h for 2 h; Dex + L-PRO group: P7 rats were administered an intraperitoneal injection of 75 *μ*g/kg Dex for five consecutive days and tail vein injection of PRO 5 mg/kg for anesthesia, followed by maintenance anesthesia at a dose of 20 mg/kg/h for 2 h in the first day. The animals were routinely fed for 30 days (P30) before the experiment.

### 2.2. Morris Water Maze Test

The Morris water maze is a round pool with a white inner wall, 150 cm in diameter and 60 cm in height. The depth of water injection in the pool is 50 cm, the temperature is 24–26°C, and the pool is divided into 4 quadrants labeled with different markers. After the last treatment, the rats were trained continuously for 4 days, and they were placed in a water maze without a platform for adaptive training, allowing them to swim freely in the water maze for 120 s. Then the rats were taken out and wiped clean to reduce the effects of scratching and the water environment, and other factors. Subsequently, a positioning navigation experiment was performed, in which the rats were randomly placed in a quadrant facing the pool wall, and the time to find the platform (escape latency) was recorded, and the recording was stopped after boarding the platform for 10 s. If the rats failed to find the platform within 120 s, they were guided onto it for 10 s and then removed, once in the morning and once in the afternoon, for 4 days. Formal experiments were performed since day 5, and escape latency, the number of crossing points across the platform quadrant, time spent in the target quadrant, swimming route, as well as swimming time were recorded. Swimming speed was measured using the formula: swimming speed = swimming distance/swimming time.

### 2.3. Passive Avoidance Test

At the end of 30 days of passive avoidance testing, each rat underwent three passive avoidance training experiments. The XBA-2 rat dark program automatic controller consists of a dark room and a light room with channel connections with electric shocks in the dark chamber provided. Latency to enter the dark compartment (step-through latency, STLr) was recorded by computer, as well as the time of returning to the light compartment after the shock recorded as the number of errors. STLr was recorded for acquisition experiments and retention experiments, and the time spent in the dark chamber (TDC) for retention experiments.

### 2.4. Toluidine Blue (Nissl) Staining

Three rats in each group were perfused and fixed with 4% paraformaldehyde, and the whole brain tissue was removed and fixed for 24 h. Coronal sections of the temporal lobe corresponding to the whole brain region were cut into sections (20 *μ*m thick). The sections were placed in 0.1 M phosphate-buffered saline (PBS) containing 0.05% sodium azide (NaN3) at 4°C, shook six times, dehydrated with gradient alcohol, and stained with Nissl staining kit (C0117, Biyuntian, Shanghai, China) at 37°C for 20–30 min. After twice washing with distilled water for 2 s each time, 95% ethanol for 3–5 s, and absolute ethanol for 1 min, the sections were dried and mounted with neutral resin. The samples were stained with Nissl and photographed and observed under a microscope with measurement of Nissl-positive neural cells in the rat hippocampus.

### 2.5. Terminal Deoxynucleotidyl Transferase-Mediated dUTP In Situ Incision End Labeling (TUNEL) Staining

The films made in step 2.4 were routinely dewaxed and dehydrated, treated with 3% hydrogen peroxide (H_2_O_2_), digested with proteinase K (20 mg/ml) for 20 min, rinsed with phosphate-buffered saline solution (PBS), and TUNEL reaction solution was added to them (C1088, Beyotime, Shanghai, China) in a humidified box at 37 °C for 1 h. Then the sample was rinsed with PBS three times, added with 50 *μ*l POD conversion agent for 30 min at 37 °C and developed with 50∼100 *μ*l DAB for 10 min, rinsed again, and sealed with neutral gum after transparency to collect images.

### 2.6. ELISA Test

The hippocampal tissues were separated from the rat brain and then added with PBS buffer solution. After homogenization, the rats were centrifuged at 4°C at 12,000 r/min for 30 min with the supernatant collected. The levels of interleukin 1*β* (IL-1*β*), IL-6, IL-10, and tumor necrosis factor (TNF-*α*) in the hippocampal tissues of rats in each group were measured in accordance with the instructions of ELISA detection kits (Jiancheng, Nanjing, China).

### 2.7. Determination of ROS, MDA, SOD, and GSH Oxidation Parameters

Rat hippocampal tissues were fully homogenized with PBS buffer and centrifuged at 12,000 r/min for 30 min at 4°C, and the upper supernatant was taken. The levels of ROS (Reactive Oxygen Species Assay Kit, CA1410), MDA (Micro Malondialdehyde Assay Kit, BC0025), SOD (Superoxide dismutase activity detection kit, BC0170), and GSH (Micro Reduced Glutathione Assay Kit, BC1175) were measured by biochemical testing kits of Solaibao Company in Beijing.

### 2.8. qRT-PCR

Total RNAs were extracted from the brain tissues of rats in each group by the TRizol method (Invitrogen, California, USA), followed by NanoDrop 2000 (Thermo Scientific, Massachusetts, USA) to detect the concentration and purity of RNA. RNA was reversely transcribed into cDNA with a RevertAid RT Kit and primers (K1691, Thermo, Massachusetts, USA). The expression levels of brain-derived neurotrophic factor (BDNF), receptor tyrosine kinase B (TrkB), and neurotrophin-3 (NT-3) mRNA were detected according to the instructions of the SYBR GREEN testing kit (TaKaRa, Kyoto, Japan). *β*-Actin was used as an internal reference control, and six replicates were set up in the experiment. The experimental data obtained by qRT-PCR were used to calculate the relative expression of the target gene by the 2^−ΔΔCt^ method, and the primer sequences are shown in Table 1.

### 2.9. Western Blot

50 *μ*g of sheared rat hippocampal tissue was placed in a centrifuge tube and mixed with 500 *μ*l of RIPA lysate (BL504 A, Biosharp, Anhui, China) containing 1 mM phenylmethylsulfonyl fluoride (PMSF) and centrifuged at 4°C, 12,000 r/min for 10 min with the supernatant collected as total protein. Protein concentration was determined with a BCA kit (23250, Thermo Fisher, Massachusetts, USA). 20 *μ*g of denatured protein was separated by 10% SDS-PAGE gel and then transferred to a polyvinylidene fluoride (PVDF) membrane, and blocked with 5% skim milk powder. The membrane was probed with primary antibodies (as shown in Table 2) overnight at 4°C and then incubated with secondary antibodies (horseradish enzyme-labeled goat antirabbit IgG (*H* + *L*), ZB2301, Zsbio, Beijing, China) for 1 h at room temperature. ECL Plus Hypersensitive Luminescent Solution (PE0010, Solarbio, Beijing, China) was used to expose and acquire bands in a gel imager, and *β*-actin was used as an internal reference for immunoblotting. Band gray values were analyzed with ImageJ software.

### 2.10. Statistical Methods

All data were expressed as mean ± standard deviation (SD), and one-way analysis of variance was performed using SPSS 24.0, with *p* < 0.0 as the significant ifferences.

## 3. Results

### 3.1. Dexmedetomidine Combined with Low-Dose Propofol Can Improve the Spatial Learning and Memory Ability of Rats

To identify the differences in the effects on spatial learning and memory ability between Dex with low-dose PRO and PRO alone, we performed a water maze test. The lipid group and the sham group shared similar escape latency, the number of platform crossings, the time spent to reach the target quadrant, and the swimming speed, excluding the effect of lipid emulsion injection on the state of the rats. On days 1–3, escape latency of the PRO and Dex + L-PRO groups was significantly longer than that of the sham group, it also declined over time, and especially the difference between the PRO and Dex + L-PRO group became more prominent by day 4 with shorter latency in the complicated group (Figure 1(a), *p* < 0.01). In addition, the number of crossing points and the time spent to reach the target quadrant decreased after PRO treatment, but the addition of L-PRO largely increased the number as well as the time (Figures 1(b) and 1(c)). Interestingly, the results showed no significant difference in the mean swimming speed among the four groups (Figure 1(d)). The above results suggested that the combination of Dex and low-dose PRO could better alleviate spatial learning and memory impairment in rats than PRO alone, with no significant difference compared with normal rats.

### 3.2. Dexmedetomidine Combined with Low-Dose Propofol Improved Passive Avoidance Test Performance in Rats

The stimulus-response behavior of the rats in each group was further evaluated using the passive avoidance test. The acquired experiment did not indicate any significant STLr among the four groups of rats (Figure 2(a)). In the retention experiment, STLr was significantly decreased and TDC was significantly increased in the L-PRO group compared with the sham group. However, the combination with Dex and PRO restored the TDC and STLr (Figures 2(b) and 2(c)).

### 3.3. Dexmedetomidine Combined with Low-Dose Propofol Attenuates Neural Cell Damage in Rat Hippocampus

Nissl staining was then conducted to assess the hippocampal nerve tissue. The results showed that the cells in the CA1 region of the Sham group and Lipid group were neatly arranged and tight, with abundant Nissl bodies observed in the cytoplasm. Meanwhile, we noticed disordered arrangement and loss of cells as well as neuronal damage in the CA1 region in the L-PRO group and Dex + L-PRO group. In the L-PRO, the cells were more loosely arranged and had obvious neuronal damage and loss with more neurons. From the above, it can be seen that the combination with Dex and PRO may alleviate the neural cell damage in rat hippocampus (Figures 3(a) and 3(b)).

### 3.4. Dexmedetomidine Combined with Low-Dose Propofol Induces Lower Apoptosis Rate in Rat Hippocampus

Han et al. held that a high dose of PRO could induce neuronal apoptosis in the developing rat brain [14], so we further studied the apoptosis of hippocampal cells in each group. TUNEL staining results depicted that apoptotic cells were significantly increased in the hippocampus of the PRO and Dex + L-PRO groups compared with that of the sham group; actually, administration of Dex based on PRO treatment has decreased the amount of apoptotic cells in the hippocampus (Figure 4(a)).

Western blot further detected the expression of apoptotic proteins cleaved caspase-3, Bcl-2, and Bax. Anesthesia with PRO alone or Dex plus L-PRO was associated with decreased expression of Bcl-2 and increased expression of Bax and cleaved caspase-3 compared with the Sham group. However, compared with L-PRO group, Dex + L-PRO group showed a higher expression of Bcl-2 and lower protein expression level of Bax and cleaved caspase-3 (Figures 4(b) and 4)(c). It shows that DEX can promote the expression of Bcl-2 protein and inhibit the expression of Bax protein and cleaved caspase-3 protein in the process of nerve injury. These results indicate that Dex combined with low-dose PRO can inhibit apoptosis PRO-induced in the rat hippocampus.

### 3.5. Dexmedetomidine Combined with Low-Dose Propofol Reduces Inflammation in the Hippocampus of Rats

Using ELISA, we continued to check up the level of inflammatory factors in the hippocampus of rats. Compared with the sham group, the levels of proinflammatory cytokines IL-1*β*, IL-6, and TNF-*α* were significantly increased in PRO and Dex + L-PRO groups, while the levels of anti-inflammatory cytokine IL-10 decreased in PRO and Dex + L-PRO groups. The advent of Dex actually mitigated the impact caused by PRO, down-regulating the levels of IL-1*β*, IL-6, and TNF-*α*, and up-regulating the levels of IL-10 (Figures 5(a)–5(d)). These results suggest that Dex combined with low-dose PRO can reduce the inflammatory response induced by dexamethasone in the rat hippocampus.

### 3.6. Dexmedetomidine Combined with Low-Dose Propofol-Induced Lower Levels of Oxidative Stress in Rat Hippocampus

In addition, we measured the substance secretion and enzyme activity in the oxidative stress response in the hippocampus of rats after anesthesia. Treatment with PRO results in elevation of ROS and MDA and decline in SOD and GSH. Importantly, addition of Dex to L-PRO greatly decreased the levels of ROS and MDA and restored the levels of SOD and GSH (Figures 6(a)–6(d)).

### 3.7. Dexmedetomidine Combined with Low-Dose Propofol Have Higher Expression of BDNF, TrkB, and NT-3

Neurotrophic factors BDNF, NT-3, and their receptor TrkB provide nutritional support for afferent sensory neurons in the inner ear [15, 16]. Therefore, we examined BDNF and NT-3 in the hippocampal tissue of rats in each group. Using RT-qPCR (Figures 7(a)–7(c)) and Western blot (Figures 7(d) and 7(e)), we found lower expression of BDNF, TrkB, and NT-3 in the hippocampus of rats in the PRO and Dex + L-PRO group relative to Sham group, with Dex greatly restored their expressions in Dex + L-PRO group.

### 3.8. Combined Regimen Can Inhibit the Activation of MAPK Pathway

Finally, we further explored the mechanism underlying the role of Dex combined with low-dose PRO in the rat hippocampus. As revealed by Western blot, the ratios of p-p38/*p*38 and p-ERK1/2/ERK1/2 in the hippocampus of rats in the L-PRO group and PRO + L-PRO group increased significantly. Meanwhile, the Dex + L-PRO group had a lower ratio of p-p38/*p*38 and p-ERK1/2/ERK1/2 than L-PRO group (Figures 8(a) and 8(b)). These results indicate that the combined regimen can inhibit the activation of the MAPK pathway induced by PRO.

## 4. Discussion

PRO is an alkylphenol derivative, chemically known as 2, 6-diisopropylphenol, which is used as a sedative and anesthetic due to its rapid onset and recovery properties [17]. However, apart from anesthesia, PRO may cause neurotoxicity by inducing neuronal apoptosis, hindering neuronal proliferation and disrupting synaptogenesis in the developing brain [18, 19]. In addition, long-term behavioral deficits in infants exposed to urea have been previously observed [20]. Therefore, the harm of PRO should be reduced when fully exerting the function in clinical practice. Previous studies have shown that Dex is safe and efficient. Schacherer et al. compared the efficiency of Dex and PRO in clinical trials and found that Dex had a higher anesthetic efficiency and a lower incidence rate of adverse events in patients, but the recovery time after PRO was significantly shorter [21]. The combination of Dex and PRO has its own different characteristics, and this study combined them and found that PRO plus DeX could significantly attenuate the nerve injury caused by PRO in developing rats and improve spatial memory ability and learning ability. These findings are consistent with those of the study by Wang et al. in rats [13]. A clinical trial of pediatric tonsillectomy reported by Tsiotou et al. demonstrated that the addition of Dex to anesthesia significantly reduces the probability and severity of delirium in patients after anesthesia [22]. It can be seen that the use of Dex in combination with low-dose PRO might reduce the harm to the patient and enhance recovery.

PRO and Dex also showed good antioxidant or anti-inflammatory activities in previous studies [23, 24]. Herein, our work noted that the combination of Dex and PRO had higher antioxidant and anti-inflammatory effects than PRO alone. Huang et al. found that the combination of dexamethasone and PRO effectively inhibits inflammation in rats with LPS-induced systemic neuroinflammation [25]. Exploring the mechanism of action of Dex, Jing et al. noted that Dex attenuated the neurotoxicity of primary hippocampal neurons through the Erk1/2/CREB/BDNF signaling pathway *in vitro* [26]. BDNF, TrkB, and NT-3 belong to brain-derived neurotrophic factors, which can control the survival, development, and function of neurons in the peripheral and central nervous systems and are closely related to the maintenance of neural cell function [27]. In the results of this study, the combination of dexamethasone and PRO significantly increased the expression of BDNF, TrkB, and NT-3, presumably by increasing the expression of brain-derived neurotrophic factor to produce a protective effect on the body. In addition, MAPK is a family of serine-threonine protein kinases, which also includes extracellular signal-regulated kinase (ERK), p38 MAPK, and c-Jun N-terminal kinase (JNK) [28]. MAPK signaling pathway plays an important role in cellular physiological and pathological processes, such as cell proliferation, differentiation, apoptosis, and stress [29]. And some studies have pointed out that the MAPK signaling pathway is involved in the regulation of the expression of BDNF, TrkB, and NT-3, and it can be seen that activation of the MAPK signaling pathway will decrease the expression of neurotrophic factors, while neurotrophic factors will also affect the activity of the MAPK signaling pathway [30]. In the results of this trial, it was found that the combination of dexamethasone and PRO significantly reduced the activity of the MAPK signaling pathway, which was supported by many relevant study results [31]. These results suggest that the combination of Dex and PRO can stimulate the expression of neurotrophic factors and protect neural cells through inhibition of the MAPK signaling pathway. Although the study indicates the protective role of Dex plus PRO in neural cell damage and learning and memory ability, there are still two limitations: (1) In this study, only a preliminary attempt was made to use Dex and low-dose PRO, and it was necessary to set up the test with different dosage ratios to obtain the optimal regimen of combination and provide more perfect test data for clinical practice. (2) The study object was limited to rats instead of human clinical evaluation, and the differences in human individuals need to be considered in practical application, so basic and clinical studies are still needed for verification.

## 5. Conclusion

Dex incorporated with low-dose PRO can reduce neuronal injury and avoid learning and memory impairment caused by anesthetics in developing rats by inhibiting inflammation, oxidative stress response, and neuronal apoptosis. The combination of Dex and low-dose PRO inhibits MAPK signaling pathway activity and promotes the secretion of nerve factors in the rat hippocampus with efficiency and safety, and thereby, this protocol shows promising potential for clinical application.

## Figures and Tables

**Figure 1:** Dexmedetomidine combined with low-dose propofol improved learning ability, memory, and motor ability in rats. (a) Escape latency of rats in each group during the water maze test; (b) number of times of the rats in each group crossed the intersection of the platform quadrant; (c) time taken for rats in each group to reach the target quadrant; (d) average swimming speed of rats in each group; ^∗∗^*p* < 0.01 vs. Sham group, ^##^*p* < 0.01*vs*. L-PRO group.

**Figure 2:** Dexmedetomidine combined with low-dose propofol improved passive avoidance test performance in rats. (a) The STLr of the acquired experiment of rats in each group; (b) the STLr of the retention experiment in each group; (c) TDC of rats in each group, ^∗∗^*p* < 0.01 vs. Sham group, ^##^*p* < 0.01 vs. L-PRO group. STLr, step-through latency; PRO, propofol; TDC, time spent in the dark chamber.

**Figure 3:** Evaluation of pathological damage of neural cells in the hippocampus of rats by Nissl staining. (a) Nissl staining was used to detect the pathological staining of neural cells in the rat hippocampus; green arrows represent stained nerve cells. (b) Quantification of the number of Nissl bodies in the hippocampus of rats in different groups in Nissl staining. ^∗∗^*p* < 0.01 vs. Sham group, ^##^*p* < 0.01*vs*. L-PRO group.

**Figure 4:** Effect of dexmedetomidine combined with low-dose propofol on apoptosis in the rat hippocampus. (a) TUNEL staining was used to observe the apoptosis in the hippocampus of rats in each group; (b) western blot was used to detect the expression of apoptosis-related proteins (cleaved caspase-3, Bcl-2, and Bax) in the hippocampus of rats in each group, ^∗∗^*p* < 0.01 vs. sham group, ^##^*p* < 0.01*vs*. L-PRO group.

**Figure 5:** Secretion levels of inflammatory factors in the hippocampus of rats in different groups. (a–d) The secretion levels of IL-1*β* (a), IL-6 (b), TNF-*α* (c), and IL-10 (d) in rat hippocampus were measured by ELISA, ^∗∗^*p* < 0.01 vs. Sham group, ^##^*p* < 0.01*vs*. L-PRO group.

**Figure 6:** Measurement of oxidative stress secretion and enzyme activity in the hippocampus of rats in different groups. (a–d) The levels of ROS (a), MDA (b), SOD (c), and GSH (d) in the hippocampus of rats in different groups, ^∗∗^*p* < 0.01 vs. Sham group, ^##^*p* < 0.01 vs. L-PRO group.

**Figure 7:** Expression of BDNF, TrkB, and NT-3 in the hippocampal tissue of rats in each group. (a–c) The mRNA expression levels of BDNF (a), TrkB (b), and NT-3 (c) in rat hippocampal tissues were detected by qRT-PCR; (d, e) the protein expression of BDNF, TrkB, and NT-3 in rat hippocampal tissues was detected by Western blot, ^∗∗^*p* < 0.01 vs. Sham group, ^##^*p* < 0.01 vs. L-PRO group.

**Figure 8:** Detection of MAPK signaling pathway protein expression levels in the hippocampus of rats in each group. (a, b) Western blot was used to detect the expression of p-p38, p38, p-ERK1/2, and ERK1/2 proteins in the MAPK signaling pathway in rat hippocampus, ^∗∗^*p* < 0.01 vs. sham group, ^##^*p* < 0.01*vs.* L-PRO group.

**Table 1:** Primer sequences for qRT-PCR.

Gene	Sequences (5′ to 3′)
BDNF	F : GGCTGACACTTTTGAGCACGTC
	R : CTCCAAAGGCACTTGACTGCTG

TrkB	F : ACAGTCAGCTCAAGCCAGACAC
	R : GTCCTGCTCAGGACAGAGGTTA

NT-3	F : CTACTACGGCAACAGAGACGCT
	R : CTACTACGGCAACAGAGACGCT
	F : GGCATCACACTTTCTACAACG

*β*-Actin	R : GGCAGGAACATTAAAGGTTTC
	R : GGCAGGAACATTAAAGGTTTC

**Table 2:** Primary antibodies used in this study.

Primary antibodies	Catalogue number	Company
BDNF	ab205067	Abcam, Cambridge, UK
TrkB	4603	Cell Signaling Technology, Boston, USA
NT-3	ab53685	Abcam, Cambridge, UK
*β*-Actin	ab8226	Abcam, Cambridge, UK
p38	8690	Cell Signaling Technology, Boston, USA
p-P38	9216	Cell Signaling Technology, Boston, USA
p-ERK1/2	9101	Cell Signaling Technology, Boston, USA
ERK1/2	9102	Cell Signaling Technology, Boston, USA
Bcl-2	ab196495	Abcam, Cambridge, UK
Bax	ab182734	Abcam, Cambridge, UK
Cleaved caspase-3	9661	Cell Signaling Technology, Boston, USA
Caspase-3	ab184787	Abcam, Cambridge, UK

## Data Availability

The data used to support the findings of this study are available from the corresponding author upon request.
